The article "Spatial variations in the biochemical potential of okra [Abelmoschus esculentus L. (Moench)] leaf and fruit under field conditions" was retracted in 2022. Reasons: compromised peer review; a conflict of interest; concerns about the authorship.

# Spatial variations in the biochemical potential of okra [*Abelmoschus esculentus* L. (Moench)] leaf and fruit under field conditions

**DOI:** 10.1371/journal.pone.0259520

**Published:** 2022-02-03

**Authors:** Samreen Sarwar, Nudrat Aisha Akram, Muhammad Hamzah Saleem, Sadia Zafar, Suliman Mohammed Alghanem, Muyassar H. Abualreesh, Aishah Alatawi, Shafaqat Ali

**Affiliations:** 1 Department of Botany, Government College University, Allama Iqbal Road, Faisalabad, Pakistan; 2 College of Plant Science and Technology, Huazhong Agricultural University, Wuhan, China; 3 Department of Botany, Division of Science and Technology, University of Education, Faisalabad, Pakistan; 4 Biology Department, Faculty of Science, Tabuk University, Tabuk, Saudi Arabia; 5 Department of Marine Biology, Faculty of Marine Sciences, King Abdualaziz University, Jeddah, Saudi Arabia; 6 Department of Environmental Sciences and Engineering, Government College University, Faisalabad, Pakistan; 7 Department of Biological Sciences and Technology, China Medical University, Taichung, Taiwan; Bangabandhu Sheikh Mujibur Rahman Agricultural University, BANGLADESH

## Abstract

Okra (*Abelmoschus esculentus* L. (Moench) plays a significant role in humans nutrition because its fresh leaves, stems, flowers, pods and seeds, are used for multiple purposes. The present study attempted to determine the spatial variations in biochemical attributes of osmoprotectants and the oxidative defense system of okra plants. Samples of soil and okra plants (leaves and fruits) were collected from three different locations: Faisalabad region-1 (7 JB-I), Faisalabad region-2 (7 JB-II) and Pindi Bhattian. Chlorophyll contents, glycine betaine (GB), ascorbic acid (AsA), total phenolics, hydrogen peroxide (H_2_O_2_), proline, and malondialdehyde (MDA) contents were analyzed in the leaves and fruits of okra plants. Soil analyses showed that pH, electrical conductivity (EC), phosphorus (P), potassium (K), iron (Fe), and saturation of soil were higher in Faisalabad region 2, while organic matter, sand, Zn, and Cu were higher in the Pindi Bhattian region. The results from okra leaves showed that Pindi Bhattian had higher chlorophyll *a*, GB and H_2_O_2_ contents, while Faisalabad region 1 had a higher ratio of chlorophyll *a*/*b* compared to the other regions. However, Faisalabad regions 2 and 1 had higher leaf phenolic contents, Faisalabad regions 1 and 2 showed higher leaf proline contents, and Faisalabad region 2 possessed higher AsA and MDA contents. Analyses of okra fruits showed that Faisalabad region 2 had higher chlorophyll *a* and total chlorophyll contents, while Faisalabad region 1 had higher chlorophyll *b* contents. Faisalabad region 2 and Pindi Bhattian had higher ratios of chlorophyll *a*/*b*, and Faisalabad region 1 showed higher phenolic, AsA, H_2_O_2_, and MDA contents of okra fruit, whereas the Faisalabad regions exhibited higher proline and GB contents than the Pindi Bhattian region. Overall, okra leaves and fruits showed better responses in the Faisalabad regions, and these results may be used to screen for okra cultivars with better tolerance under different environmental conditions.

The article "Spatial variations in the biochemical potential of okra [Abelmoschus esculentus L. (Moench)] leaf and fruit under field conditions" was retracted in 2022. Reasons: compromised peer review; a conflict of interest; concerns about the authorship.

## 1. Introduction

Okra is considered a high-value nutraceutical vegetable crop that is grown in different regions around the globe [1–3]. It is a great source of nutrients that are necessary for multiple purposes of human health [4, 5]; Durazzo et al. [6]. Okra seeds are a good source of proteins and in human diet, proteins play a significant role in balancing nutrition [7]. The main health benefit of okra is its capacity to manage cholesterol level in the human body. Therefore, it is helpful for weight loss and reducing cholesterol to maintain a healthy and strong body [8]. Due to these qualities, okra is seen as beneficial by diet consultants [9], beneficial for asthma patients, and normalizes cholesterol and blood sugar [1]. It has the ability to bind bile acids to control cholesterol and protect against cancer. Its seeds prevent diabetes by maintaining blood glucose [6, 10].

Plant and soil community composition, nutrient availability and species interactions are altering due to changes in climate [11–16]. However, there is a lack of knowledge regarding how environmental factors can cause alterations [17–21]. Changes in developmental routes occur in plants due to their genetic diversity and the varying ecological states in which species emerge. Within a plant, environmental variations have different consequences on varying tissues and organs at the cellular, molecular, morphological levels, and reproductive levels of a plant [22–26]. Normally, aerobic metabolism continually produces reactive oxygen species (ROS) that restrict numerous components of the plant [27–32]. Under favorable conditions, ROS are continually produced at a basal level. Moreover, if they are scavenged by several antioxidant mechanisms, they are able to minimize damage [33–36]. Therefore, the survival of plants depends on several factors, such as severity, variation in growth conditions and capability to adopt the environment [37–40]. The ubiquitous nature of the antioxidant machinery triggers the need for detoxification of ROS for cellular survival [41–46]. Hydrogen peroxide is generated in plant cells by oxidative stress, which is produced by different factors, such as UV radiation, wounding, drought, pathogen infection, salinity, chilling and intense light [47–50]. Proline is an osmolyte that acts as a nonenzymatic antioxidant and is widely used to combat the harmful effects of many ROS members. Proline accumulates in plants during stress in significant amounts and is a stress tolerance indicator [51–56].

The article "Spatial variations in the biochemical potential of okra [Abelmoschus esculentus L. (Moench)] leaf and fruit under field conditions" was retracted in 2022. Reasons: compromised peer review; a conflict of interest; concerns about the authorship.

Based on the above facts, the objectives of the present study were to assess the comparative account of analyses of leaf and fruit with respect to physiological and biochemical changes. Moreover, we determined the spatial variations in chlorophyll contents, osmoprotectants, and oxidative defense system of okra leaf and fruit.

## 2. Materials and methods

The samples of okra leaves and fruits were collected from three different locations of Central Punjab, Pakistan i. e., Faisalabad regions (two different locations) and Pindi Bhattian.

The “Faisalabad and Pindi Bhattian” longitude 73.06° E, latitude 31.26° N and elevation of 184.5 m from mean sea level. The weather conditions during the study period preseted in Table 1. These three locations are property of a local farmer and were already widely used for the cultivation of okra at commercial level. So, we collected samples with permission of farmer without involvement of any ethical committee. The climate of central and southern Punjab possesses the dry semi-arid agro-climatic properties. These regions has good canal irrigation system so included in productive agriculture zones. The spatial variations were confirmed by soil analyses. Soil samples were collected from four different sites of each of three locations and analyzed at the Ayub Agricultural Research Institute, Faisalabad, Pakistan and data collected presented in Table 2. Ethical approval was taken from Department Ethical Review Committee to conduct study and no plants or experiments was harmed in this study. From each location, four sites were selected The collected leaf and fruit samples were analyzed to determine the following different physiological and biochemical parameters:

**Table 1:** Meteoriologiacl average data collected from three different regions.

	Faisalabad region-I	Faisalabad region-II	Pindi Bhattian
Sun shine (h)	8.7	8.6	8.8
Temperature (°C)	31.4	31.7	30.6
Humidity (%)	65.1	66	64.2
Rain fall (mm)	41.7	38.6	39.1

**Table 2:** Different physical and chemical characteristics of soil collected from three different regions.

Soil characteristics	Faisalabad region-I	Faisalabad region-II	Pindi Bhattian
pH	7.4	7.6	7.2
EC (dS m^-1^)	1.202	1.72	1.04
Phosphorous (ppm)	2.2	4.45	2.75
Potassium (ppm)	172	215	154
Organic matter (%)	0.82	0.77	0.91
Saturation (%)	32	34	31
Sand (%)	42.4	51.7	55.4
Silt (%)	21.2	17.5	20
Clay (%)	35.3	29.6	28.9
Texture	Loam	Loam	Loam
Zn (ppm)	0.49	0.36	0.51
Iron (ppm)	2.13	2.42	2.19
Copper (ppm)	0.09	0.11	0.14

The article "Spatial variations in the biochemical potential of okra [Abelmoschus esculentus L. (Moench)] leaf and fruit under field conditions" was retracted in 2022. Reasons: compromised peer review; a conflict of interest; concerns about the authorship.

### 2.1. Chlorophyll contents

Chlorophyll *a* and *b* concentrations were determined following the method of Arnon [57]. Fresh leaf and fruit samples (0.25 g) were homogenized in 5 mL of acetone (80%). Then, samples were placed overnight at 4°C. Chlorophyll contents were measured by reading the absorbance of the supernatant using an Ultra Violet-visible spectrophotometer (Model Hitachi-U 2001) at 663 and 645 nm.

### 2.2. Glycine betaine (GB) contents

Dried fruit and leaves (0.25 g) were mixed with 0.5% toluene (10 mL) and preserved at 4°C for one day. After that, the mixture was filtered, and the filtrate (1 mL) was mixed with 2 *N* sulfuric acid (H_2_SO_4_) (1 mL) and 0.2 mL of potassium tri-iodide (KI_3_) in test tubes. This mixture was kept at 4°C for 90 min, after which 2.8 mL of deionized water and 6 mL of 1,2 dichloroethane were added to each sample. Then, discard the upper layer and absorbance of the lower layer was measured at 365 nm using a spectrophotometer following Grieve and Grattan [58].

### 2.3. Ascorbic acid (AsA) contents

Ascorbic acid (AsA) was determined following the method of Mukherjee and Choudhuri [59]. Fresh fruit and leaves (0.25 g) were homogenized with 6% trichloroacetic acid (TCA) (10 mL: w/v), and 4 mL of supernatant was mixed with 2 mL of dinitrophenyl hydrazine. One drop of 10% thiourea was added, boiled for 15 min and subsequently cooled. Then, 80% H_2_SO_4_ (5 mL) was added. The absorbance of the samples was measured at 530 nm using a spectrophotometer.

### 2.4. Total phenolic contents

Total phenolics were determined using the protocol proposed by Julkunen-Titto [60]. Fresh leaf and fruit samples (0.25 g) were ground in 80% acetone (5 mL). Then, this extract was filtered through filter paper, and 100 μL of supernatant was mixed with Folin-phenol Ciocalteus reagent (1 mL) and 2 mL of distilled water. After that, the volume was brought up to 10 mL with distilled water and 5 mL of 20% sodium carbonate (Na_2_CO_3_). Then, the estimation of total phenolics was performed at 750 nm via a spectrophotometer.

### 2.5. Hydrogen peroxide (H_2_O_2_) contents

Hydrogen peroxide contents were measured following the method proposed by Velikova et al. [61]. Fresh samples of leaf and fruit (0.25 g) were ground in a mortar and pestle along with 0.1% TCA (5 mL). Then, the samples were filtered, and 0.5 mL of phosphate buffer and 1 mL of potassium iodide were mixed with 0.5 mL of the supernatant. Subsequently, the mixture was vortexed, and the absorbance was recorded at 390 nm using a spectrophotometer.

### 2.6. Proline contents

The proline contents of leaf and fruit were determined following the protocol described by Bates et al. [62]. Fresh leaves and fruit (0.25 g) were mixed with 5 mL of sulfosalicylic acid (3% w/v). Then, the mixture was filtered, and 2 mL of filtrate was taken. The reaction mixture consisted of 2 mL of proline extract, 2 mL of ninhydrin and the addition of 2 mL of glacial acetic acid. The mixture was boiled at 95°C for 60 min. After cooling the mixture, 4 mL of toluene were added to the mixture to generate two layers. The absorbance was recorded at 520 nm using a spectrophotometer.

The article "Spatial variations in the biochemical potential of okra [Abelmoschus esculentus L. (Moench)] leaf and fruit under field conditions" was retracted in 2022. Reasons: compromised peer review; a conflict of interest; concerns about the authorship.

### 2.7. Malondialdehyde (MDA) contents

Malondialdehyde contents were determined following the method of Carmak and Horst [63]. Fresh leaf and fruit (0.25 g) were ground in 1% TCA (5 mL), and this mixture was centrifuged at 15,000 *rpm* for 10 min. Then, 0.5% TBA (thiobarbituric acid), 20% TCA and supernatant were mixed in equal volumes. This mixture was boiled for 30 min at 100°C. The optical density (OD) were measured at 600 and 532 nm using a spectrophotometer.

### 2.8. Statistical analysis

Analysis of variance (ANOVA) using a Costat program (Cohert v.3.6) was applied to assess the biochemical changes in leaf and fruit of okra plants. A completely randomized block design (CRD) with five replicates was established. For analyses of okra leaves and fruits, four locations were selected from each of three different sites. The graphical presentation was carried out by using Origin-Pro 2017.

## 3. Results

The present study was carried out to determine the comparative leaf and fruit biochemical changes in okra (*Abelmoschus esculentus*) leaves and fruits. They were collected from three different sites, namely, Faisalabad region 1 (7 JB-I), Faisalabad region 2 (7 JB-II), and Pindi Bhattian. The chlorophyll *a* content in okra leaves was significantly (*P* ≤ 0.01) different among the three different locations (Table 3). However, leaves collected from the Pindi Bhattian region showed more chlorophyll *a* content than leaves collected from Faisalabad region 1 and Faisalabad region 2 (Fig 1A). Chlorophyll *b* contents showed highly significant (*P* ≤ 0.001) differences between these three locations (Table 3). On the other hand, Faisalabad region 1 had a less significant effect on chlorophyll *b* than other regions in this study, and maximum chlorophyll *b* was observed in Faisalabad region 2 (Fig 1B). The results showed that the chlorophyll *a*/*b* ratio between Faisalabad region 1, Faisalabad region 2 and Pindi Bhattian exhibited highly significant (*P* ≤ 0.001) differences for this attribute (Table 3). Moreover, Faisalabad region 1 showed the maximum ratio of chlorophyll *a*/*b*, while the second region showed the minimum chlorophyll *a/b* ratio (Fig 1C). The data presented in Table 3 showed that there was a highly significant (*P* ≤ 0.001) difference between all three ecotypes of okra for total chlorophyll contents (Table 3). However, leaves collected from Faisalabad region 2 and Pindi Bhattian showed more significant differences than those collected from Faisalabad region-I (Fig 1D).

The article "Spatial variations in the biochemical potential of okra [Abelmoschus esculentus L. (Moench)] leaf and fruit under field conditions" was retracted in 2022. Reasons: compromised peer review; a conflict of interest; concerns about the authorship.

**Fig 1:** Physiological attributes (**A** = Chlorophyll *a***, B** = Chlorophyll *b***, C =** Chlorophyll *a/b* ratio, **D =** Total chlorophyll, **E =** Total phenolics, **F =** Leaf free proline, **G =** Glycine betaine, **H =** H_2_O_2_, **I =** Ascorbic acid, **J =** MDA) in leaves of okra (*Abelmoschus esculentus* L.) plants obtained from two regions of Faisalabad (different locations) and Pindi Bhattian.

**Table 3:** Analysis of variance of the physiological attributes of okra fruit (*Abelmoschus esculentus* L.) collected from three different regions [Faisalabad (7 JB-I, 7 JB-II) and Pindi Bhattian].

Sources	df	Chlorophyll *a*	Chlorophyll *b*	Chlorophyll *a/b*	Chlorophyll	Phenolics	Proline	Glycine betaine	Hydrogen per oxide	Ascorbic Acid	MDA
**Blocks**	**3**	3.4292ns	0.0021ns	0.0021ns	0.0025ns	0.0378ns	0.1408ns	50.553ns	13.671ns	0.0415ns	2286.4ns
**Ecotypes**	**2**	0.0852***	0.0181ns	0.6411***	0.0250ns	2.4611***	2.3851ns	177.55*	5286.8***	10.333***	16002.1**
**Error**	**6**	0.0014	0.0061	0.0030	0.0119	0.0136	0.5173	25.012	49.348	0.3416	9931.5

** = significant at 0.01 level; ns = no significant.

The total phenolic contents showed no significant difference between all three ecotypes of okra plants collected from the three different regions (Table 3). However, Faisalabad regions 2 and 1 showed greater phenolic contents than Pindi Bhattian (Fig 1E). The leaf free proline contents showed no significant variation between all three ecotypes of okra leaves (Table 3). However, Faisalabad region 1 and region 2 showed higher proline contents than Pindi Bhattian (Fig 1F). Glycine betaine contents showed a highly significant (*P* ≤ 0.001) difference between all three locations in the leaves of the okra plant (Table 3). However, leaf samples collected from Pindi Bhattian had maximum glycine betaine (Fig 1G) and hydrogen peroxide contents (Fig 1H) compared to Faisalabad samples. Hydrogen peroxide contents showed a highly significant (*P* ≤ 0.001) increase in all okra leaves from the three locations (Table 3). Analysis of variance showed that there was no significant difference in ascorbic acid of these three ecotypes (Table 3). However, Faisalabad region 2 contained high contents of ascorbic acid, followed by region 1 and Pindi Bhattian (Fig 1I). MDA contents showed no significant differences between the leaf samples collected from the three different regions (Table 3). Moreover, Faisalabad region 2 showed greater malondialdehyde contents than the other two regions (Fig 1J).

The article "Spatial variations in the biochemical potential of okra [Abelmoschus esculentus L. (Moench)] leaf and fruit under field conditions" was retracted in 2022. Reasons: compromised peer review; a conflict of interest; concerns about the authorship.

The results from okra fruits showed that chlorophyll *a* content possessed highly significant (*P* ≤ 0.001) variations for all three ecotypes (Table 3). However, Faisalabad region 2 showed better performance for chlorophyll *a* than Pindi Bhattian and Faisalabad region 1 (Fig 2A).

**Fig 2:** Physiological attributes (**A** = Chlorophyll *a*, **B** = Chlorophyll *b*, **C =** Chlorophyll *a/b* ratio, **D =** Total chlorophyll, **E =** Total phenolics, **F =** Fruit free proline, **G =** Glycine betaine, **H =** H_2_O_2_, **I =** Ascorbic acid, **J =** MDA) in okra fruit (*Abelmoschus esculentus* L.) plants obtained from two regions of Faisalabad (different locations) and Pindi Bhattian.

Fruit samples of these three locations proved that chlorophyll *b* contents had no significant effect on any of the three okra ecotypes. Maximum chlorophyll *b* contents were observed in Faisalabad region 1 compared with other okra ecotypes (Table 3 and Fig 2B). It was observed that the chlorophyll *a*/*b* ratios among fruit samples from all locations showed a highly significant difference (*P* ≤ 0.001) (Table 3). However, ecotypes of Faisalabad region 2 and Pindi Bhattian contained a higher ratio of chlorophyll *a*/*b* than Faisalabad region 1 (Fig 2C). The total chlorophyll contents in okra fruits were not significantly different (Table 3). However, the Faisalabad region 2 ecotype showed a maximum value for total chlorophyll compared to the other ecotypes (Fig 2D).

Total phenolic contents in fruits of okra plants collected from two different regions of Faisalabad and Pindi Bhattian demonstrated a highly significant (P ≤ 0.001) difference (Table 3). Furthermore, Faisalabad region 1 showed higher phenolic content than the other two regions (Fig 2I). Statistical analysis illustrated that there was no significant change in proline content between all three ecotypes of okra fruits (Table 3). However, ecotypes of Faisalabad regions contained high contents of proline compared to the Pindi Bhattian region (Fig 2F). Glycine betaine contents showed significant (P ≤ 0.05) differences between the values of this attribute for fruit samples of all three ecotypes (Table 3). However, the Faisalabad regions showed higher contents of glycine betaine than the Pindi Bhattian regions (Fig 2G). Fruit samples were obtained from three different locations for the determination of H_2_O_2_ contents. H_2_O_2_ production in okra fruits showed a highly significant difference (*P* ≤ 0.001) among all three ecotypes (Table 3). However, Faisalabad region 1 showed higher contents of H_2_O_2_ than other regions (Fig 2H). Analysis of variance indicated that ascorbic acid showed a highly significant (*P* ≤ 0.001) difference between all three ecotypes of okra fruit samples (Table 3). Moreover, Faisalabad region 1 showed a higher quantity of ascorbic acid, Faisalabad region 2 showed moderate ascorbic acid contents, and the Pindi Bhattian ecotype showed a lower content of ascorbic acid (Fig 2I). Malondialdehyde contents in fruit samples demonstrated highly significant (*P* ≤ 0.01) results among all three ecotypes (Table 3). However, more malondialdehyde contents were observed in Faisalabad region 1 than in Faisalabad region 2 and Pindi Bhattian (Fig 2J).

The article "Spatial variations in the biochemical potential of okra [Abelmoschus esculentus L. (Moench)] leaf and fruit under field conditions" was retracted in 2022. Reasons: compromised peer review; a conflict of interest; concerns about the authorship.

## 4. Discussion

Chlorophyll plays an important role in the process of photosynthesis and acts as a transitional factor in the transformation of absorbed solar energy and synthesis of organic substances in plants [64]. During the photosynthetic process, chlorophyll *a* and *b* act as photoreceptors in plants [65]. Chlorophyll provides important information about the physiological status of plants and functions as an indicator of photosynthetic processes, production, growth, development, and biochemical aspects of plant species. Chlorophyll values change with variation in growing seasons, such as sunlight, precipitation, and temperature [66]. Chlorophyll plays a significant role in photosystem protection, light harvesting, and other growth-related functions [67].

The results obtained from the present study indicated that chlorophyll contents vary significantly among all three ecotypes of okra (leaves and fruits). Previous studies suggested that temperature variations have a large influence on chlorophyll contents, although this relationship is not comparable for all previously reported species [68]. A previous study also supported the present results showing that the leaf nutrient contents of the examined species were similar or greater than those found in other earlier studies [69]. In a previous study, a positive correlation was found between leaf nitrogen and chlorophyll contents, but depending upon soil availability, these relationships may be significantly different within species [70]. Under salt stress, a variable response of chlorophyll contents has been reported for many species depending upon their ability to tolerate salt [71].

Ascorbic acid (a water-soluble vitamin) possesses antioxidant properties and acts as a coenzyme for numerous metabolic activities [72]. It was found to be the main component circulating in the leaves of *Eryngium foetidum* [73]. Data obtained from the present study showed that the ascorbic acid content in the leaves of okra was higher in the ecotype of the Faisalabad regions, while the Pindi Bhattian ecotype showed lower ascorbic acid content. The ascorbic acid contents of okra fruits were significantly increased in the Faisalabad ecotype and significantly decreased in the other ecotype (*P* ≤ 0.001). Saraswathi et al. [74] also studied the ecotypic variations in Indian populations of *E*. *foetidum* and found that ascorbic acid was comparatively significantly higher in the population of Kamataka. Significantly lower contents of ascorbic acid were observed in the Darjeeling population than in the other ecotypes. Differences in ascorbic acid contents have been studied in *Chenopodium quinoa* wild ecotypes [75].

The article "Spatial variations in the biochemical potential of okra [Abelmoschus esculentus L. (Moench)] leaf and fruit under field conditions" was retracted in 2022. Reasons: compromised peer review; a conflict of interest; concerns about the authorship.

Malondialdehyde is one of the final products of the oxidative alteration of lipids and is responsible for cell membrane injury involving alterations to the intrinsic properties of membrane-like ion transport, fluidity, and loss of enzyme activity. These changes ultimately result in cell death [76, 77]. In the present investigation, greater MDA contents in leaves of okra were observed in the ecotype of Faisalabad region 2 compared to other ecotypes because the soil had greater salinity in this ecotype. Although malondialdehyde contents in okra fruits changed significantly (P ≤ 0.001), greater MDA contents were measured in the Faisalabad-1 ecotype. Previous findings also showed that MDA content increased with increasing salinity in the roots and leaves of both cotton cultivars, indicating cell membrane injury in both cultivars of cotton. However, MDA was greater in cv. Simian 3 as compared to cv. CCRI-79, indicating a higher degree of lipid peroxidation in cv. Simian 3 because of salt stress [78]. The same findings for lipid peroxidation have been reported by other researchers in barley (*Hordeum vulgare*) [79].

Proline plays a significant role against salinity stress in plants and acts as an osmolyte. It can also play a role as a free radical scavenger, enzyme protectant, cytosolic pH buffer stabilizer for subcellular structures, and cell redox balancer [80]. The present results showed that the ecotype of Faisalabad showed higher proline content in okra leaves and fruits than those from Pindi Bhattian, and the soil of the Faisalabad ecotype had greater salinity and possessed a higher pH value than that of the Pindi Bhattian ecotype. Campos et al. [81] explained that the activities of antioxidant enzymes can also be modified by proline. Rahneshan et al. [82] studied proline contents in the roots and leaves of two pistachio cultivars, Badami-e-Sefid (BS) and Badami-Rize-Zarand (BZ), and investigated the significance differences between these cultivars. Proline contents were enhanced significantly in roots and leaves of the BZ cultivar.

The article "Spatial variations in the biochemical potential of okra [Abelmoschus esculentus L. (Moench)] leaf and fruit under field conditions" was retracted in 2022. Reasons: compromised peer review; a conflict of interest; concerns about the authorship.

The phenolic content of plants is also affected by several environmental factors, such as rainfall, soil type, and sun exposure [83]. Kumari et al. [84] studied the comparison of phenolic contents in many millet varieties, such as proso millet, finger millet and foxtail, in Sri Lanka and investigated the significant differences in total phenolic contents between finger millet varieties. The synthesis of phenolic compounds is positively affected by long sunlight exposure with high ultraviolet radiations [85], and these findings are related to the present study, which found that the total phenolic contents in okra fruits varied significantly among all three ecotypes. Greater phenolic contents were observed in the Faisalabad ecotype than in the Pindi Bhattian ecotype, but no significant changes were observed in the okra leaves of all three ecotypes.

H_2_O_2_ plays an important role in many signaling channels in plants, including stomatal responses, pathogen elicitor responses, systemic acquired resistance, and even programmed cell death [86]. The present investigation suggested that H_2_O_2_ contents significantly increased in the leaves and fruits of okra plants between all three ecotypes. The Pindi Bhattian ecotype showed greater H_2_O_2_ contents in leaves, but in fruits of okra, H_2_O_2_ production was enhanced significantly (*P* ≤ 0.001) among the Faisalabad ecotypes because the soil of this ecotype contained high EC and had a high pH value compared to the other ecotype in the present study, which is supported by previous studies. Zhang et al. [87] also studied two cotton cultivars, Simian 3 (salt-sensitive) and CCRI-79 (salt-tolerant), and found that after sodium chloride (NaCl) treatment, H_2_O_2_ contents were enhanced in the roots and leaves of cv. Simian 3 and decreased in cv. CCRI-79 because H_2_O_2_ scavenging activity was decreased in the salt-sensitive cultivar. Previous findings also showed that in the salt-tolerant rice cultivar FL 478, the H_2_O_2_ contents were significantly (*P* ≤ 0.001) enhanced as compared to cv. IR29 (salt-sensitive) under temperate saline conditions [88].

Glycine betaine acts as an osmolyte and defends plants against abiotic stresses through osmoprotection or osmoregulation. Glycine betaine plays a significant role in the protection of photosynthetic machinery, slows ROS accumulation and involved in membrane protection [89]. The present study found that glycine betaine contents vary significantly (*P* ≤ 0.05) in fruits of okra, and greater glycine betaine contents were observed in the Faisalabad ecotypes, but in leaves of okra, greater GB contents were found in the Pindi Bhattian ecotype, which showed a significant difference (*P* ≤ 0.001). Al-Hassan et al. [90] studied three species of Plantago under salt stress and found a significant difference (*P* ≤ 0.05) in glycine betaine contents among Plantago species. However, more GB contents were observed in *P*. *coronopus* than in *P*. *major* because this species was salt sensitive. The GB contents were not increased significantly in this species, and the K^+^ concentration decreased only at concentrations above 400 mM NaCl, while in P. *coronopus*, the concentration of K^+^ decreased at moderate salinity level.

The article "Spatial variations in the biochemical potential of okra [Abelmoschus esculentus L. (Moench)] leaf and fruit under field conditions" was retracted in 2022. Reasons: compromised peer review; a conflict of interest; concerns about the authorship.

## 5. Conclusion

The soil was better in Faisalabad region 2, and overall, chlorophyll contents and glycine betaine, ascorbic acid, total phenolics, H_2_O_2_, proline, and MDA contents were higher in leaves and fruits of the okra plant of Faisalabad regions. Thus, okra leaves and fruits had better resistance in Faisalabad regions. Therefore, these findings could be used for the cultivation of okra in Faisalabad region for better tolerance under different environmental stresses.

## Supporting information

S1 Graphical abstract (TIFF)
